# Effects of Downregulation of MicroRNA-181a on H_**2**_O_**2**_-Induced H9c2 Cell Apoptosis via the Mitochondrial Apoptotic Pathway

**DOI:** 10.1155/2014/960362

**Published:** 2014-02-11

**Authors:** Lei Wang, He Huang, Yang Fan, Bin Kong, He Hu, Ke Hu, Jun Guo, Yang Mei, Wan-Li Liu

**Affiliations:** ^1^Department of Cardiology, Renmin Hospital of Wuhan University, Jiefang Road 238, Wuhan 430060, China; ^2^Cardiovascular Research Institute of Wuhan University, Jiefang Road 238, Wuhan 430060, China

## Abstract

Glutathione peroxidase-1 (GPx1) is a pivotal intracellular antioxidant enzyme that enzymatically reduces hydrogen peroxide to water to limit its harmful effects. This study aims to identify a microRNA (miRNA) that targets GPx1 to maintain redox homeostasis. Dual luciferase assays combined with mutational analysis and immunoblotting were used to validate the bioinformatically predicted miRNAs. We sought to select miRNAs that were responsive to oxidative stress induced by hydrogen peroxide (H_2_O_2_) in the H9c2 rat cardiomyocyte cell line. Quantitative real-time PCR (qPCR) demonstrated that the expression of miR-181a in H_2_O_2_-treated H9c2 cells was markedly upregulated. The downregulation of miR-181a significantly inhibited H_2_O_2_-induced cellular apoptosis, ROS production, the increase in malondialdehyde (MDA) levels, the disruption of mitochondrial structure, and the activation of key signaling proteins in the mitochondrial apoptotic pathway. Our results suggest that miR-181a plays an important role in regulating the mitochondrial apoptotic pathway in cardiomyocytes challenged with oxidative stress. MiR-181a may represent a potential therapeutic target for the treatment of oxidative stress-associated cardiovascular diseases.

## 1. Introduction

Growing evidence demonstrates that increased levels of reactive oxygen species (ROS) are associated with a variety of cardiovascular diseases [1]. Although ROS can originate from different organelles, mitochondria are considered to be the main producers of ROS. Approximately 80% of anion superoxide (O_2_^•^) is produced by mitochondria [2]. In the heart, approximately 30% of the total volume is occupied by mitochondria, and thus the heart is easily subjected to oxidative damage by ROS [3]. To combat the deleterious effects of ROS, mitochondria have evolved an intrinsic antioxidant defense network that mainly consists of the superoxide dismutase (SOD), NADH, and a complete glutathione redox system, formed by glutathione reductase, reduced glutathione (GSH), and glutathione peroxidase (GPx) [4].

GPx converts H_2_O_2_ and lipid hydroperoxides into water, using GSH as an electron donor. GPx1 is the main isoform, produced in all tissues and expressed in both the cytosol and the mitochondrial matrix. GPx1 prevents the formation of the highly reactive hydroxyl radical [5]. Several genetically modified animal models have been used to show the protective role of GPx1 in cardiac damage caused by ischemia-reperfusion injury [6–8]. Recent findings also indicate that the lack of GPx1 contributes to the risk of atherosclerosis and cardiovascular disease. Mice deficient in GPx1 (GPx1^−/−^/ApoE^−/−^) developed significantly more atherosclerosis than the control apolipoprotein E-deficient mice [9, 10]. Additionally, transgenic mice overexpressing Gpx1 were protected from aging-related enhanced susceptibility to venous thrombosis compared with wild-type mice [11]. Gpx1 also plays a pivotal role in the protection against angiotensin II-induced vascular dysfunction [12].

The posttranscriptional regulation of GPx1 expression in oxidative stress via nuclear factor *κ*B (NF*κ*B) and activator protein 1 (AP-1) has been shown by many investigators [13, 14]. However, the posttranscriptional mechanism of Gpx1 in response to H_2_O_2_-mediated oxidative stress in cardiomyocytes has not been thoroughly studied. MicroRNAs (miRNAs) are one example of a translational mechanism for the regulation of a large number of developmental and physiological processes in the heart [15]. An miRNA is a small, single-stranded RNA that is approximately 22 nucleotides (nt) long. miRNAs are widely distributed and induce both messenger RNA (mRNA) degradation and the suppression of protein translation based on sequence complementarity between the miRNA and its target [16].

The H9c2 rat cardiomyocyte cell line was chosen in the present study as this cell line retains the characteristics of isolated primary cardiomyocytes [17]. We investigated the role of miR-181a in regulating H9c2 cell apoptosis and modulating the mitochondrial apoptotic pathway in the setting of oxidative stress. We found that miR-181a is upregulated in cardiomyocytes with oxidative stress and that the downregulation of miR-181a significantly inhibited the H_2_O_2_-induced cellular apoptosis, ROS production, mitochondrial structure disruption, and activation of key signaling proteins in the mitochondrial apoptotic pathway. These protective effects were mediated at least partially through the direct targeting of Gpx1.

## 2. Materials and Methods

### 2.1. Cell Culture and Determination of Cell Viability

HEK293 cells, myogenic L6 cells, and H9c2 cells (from the Cell Bank of the Chinese Academy of Sciences, Shanghai, China) were cultured in Dulbecco's modified Eagle's medium (DMEM, Invitrogen) supplemented with 5 g/L glucose and 15% (v/v) fetal bovine serum. The cells were maintained in a humidified 37°C incubator with 5% CO_2_, supplied with fresh medium every 3 days, and subcultured before reaching confluence. The H9c2 cells were seeded in 96-well microtiter plates and treated with different concentrations of H_2_O_2_ for 2 h. The MTT assay was used to determine cell viability, following the manufacturer's protocols.

### 2.2. Bioinformatics Analysis

Rat Gpx1 3′ untranslated region (3′ UTR) sequences were retrieved from the Entrez Nucleotide database (http://www.ncbi.nlm.nih.gov/nuccore). Potential miRNAs targeting Gpx1 were predicted by miRDB (http://mirdb.org/miRDB/), TargetScan (http://www.targetscan.org/), and MicroRNA.ORG (http://www.microrna.org/).

### 2.3. Transfections, Constructs, and Dual Luciferase Reporter Assay

HEK293 and H9c2 cells were transfected with 50 nM mature miR-181a and miR-CTL (GuangzhouRuiBio Corp., Guangzhou, China) using Lipofectamine 2000 (Invitrogen, USA) as previously described [18]. H9c2 cells were also transfected with a final concentration of 100 nM and for miR-181a knockdown anti-miR-181a (Guangzhou RiBo Corp., Guangzhou, China). The anti-CTL and anti-miR-181a are represented as the scrambled inhibitor and miR-181a inhibitor, respectively. The anti-miR-181a contained 2′-OMe modifications at every base.

The 3′ UTR of the Gpx1 gene was amplified by PCR from total RNA extracted with a Genomic DNA Extraction kit (TaKaRa Bio Inc., Tokyo, Japan) from myogenic L6 cells. The sequences of the primers for the Gpx1 3′ UTR and mutant Gpx1 3′ UTR were as follows: R-Gpx1-3′ UTR-F, CCG**CTCG AG**CCTAAGGCATTCCTGGTATCTGG; R-Gpx1-3′ UTR-R, GAAT**GCGGCCG C**TTCTTTGACATTCAGCACTTTATTC; and R-Gpx1-3′ UTR-Mut-R, GAAT**GCGGC CGC**TTCTTTG**AGAATGA**GCACTTTATTCTTAG. The bold letters in the primers indicate XhoI and SalI restriction sites. The PCR products were excised with XhoI and NotI and cloned into the pmiR-RB-REPORT vector (GuangzhouRuiBio Corp., Guangzhou, China). This plasmid contains hRluc (synthetic renilla luciferase gene), encoding renilla luciferase as the reporter, and hluc (synthetic firefly luciferase gene), encoding firefly luciferase as the internal control. The recombinant plasmid pmiR-RB-Gpx1-3′ UTR was confirmed by restriction enzyme digestion and DNA sequencing.

The luciferase assays were performed according to the manufacturer's protocol. HEK293 cells, seeded into 96-well plates at a density of 1.5 × 10^4^ per well, were transfected with pmiR-RB-Gpx1-WT-3′ UTR (100 ng/well), pmiR-RB-Gpx1-Mut-3′ UTR (100 ng/well), mature miR-181a (50 nM), or miR-control (50 nM) using Lipofectamine 2000. Forty-eight hours after-transfection, the cells were lysed and assayed for luciferase activity using the Dual Glo Luciferase Assay System (Promega). Data recorded by the luminometer were normalized by dividing the firefly luciferase activity with the renilla luciferase activity.

### 2.4. Measurement of Lactate Dehydrogenase (LDH) and Malondialdehyde (MDA) Levels

H9c2 cells were transfected with miRNAs for 6 h and cultured for 24 h. H_2_O_2_ (400 µM) was added for the last 2 h. Subsequently, the cells were harvested and lysed. LDH release and MDA content were measured using commercial kits (Jiancheng Bioengineering Institute, China), according to the manufacturer's instructions.

### 2.5. Intracellular Reactive Oxygen Species (ROS) Assay

H9c2 cells were grown to confluence in a 96-well plate and then transfected with miRNAs for 6 h and cultured for 24 h. H_2_O_2_ (400 µM) was added for the last 2 h. The cells were then incubated with 2′,7′-dichlorofluorescin-diacetate (DCFH-DA, Sigma) at 37°C for 30 min. The DCFH-DA stain detecting ROS production was observed using a fluorescence microscope (Nikon, Japan). Fluorescence was read at 485 nm for excitation and 530 nm for emission with an Infinite M200 Microplate Reader (Tecan, Switzerland).

### 2.6. Annexin V and PI Binding Assay

The Annexin V and PI Fluorescein Staining kits (Bender MedSystems, Austria) were utilized to measure H9c2 cell apoptosis, according to the manufacturer's instructions. Briefly, a single-cell suspension was prepared and cultured in a six-well plate at a density of 1 × 10^5^/well. Twenty-four hours after transfection, cells from each group were collected and resuspended in two hundred microliters of 1x binding buffer. The cells were then incubated with annexin V (1 : 20) for 3 min followed by incubation with propidium iodide (PI, 1 mg/mL) for 15 min. The apoptosis rate was evaluated by flow cytometry (BD).

### 2.7. Measurement of Mitochondrial Membrane Potential

H9c2 cells were grown on cover slips and incubated with 5 µg/mL JC-1 dye (Enzo Life Sciences, USA) at 37°C for 30 min. The cells were analyzed immediately with a fluorescence microscope. JC-1 accumulates in the mitochondria, selectively generating an orange J-aggregate emission profile (590 nm) in healthy cells. However, upon cell injury, the membrane potential decreases, and JC-1 monomers are generated, resulting in a shift to green emission (529 nm). The orange and green fluorescence intensities were detected using an Infinite M200 Microplate Reader. The Δ*ψ*m of the H9c2 cells in each treatment group was calculated as the ratio of orange to green fluorescence and expressed as a multiple of the level in the control group.

### 2.8. Quantitative Real-Time PCR

Total RNA was extracted from H9c2 cells using the Trizol Reagent (Invitrogen). The RT primers and primer sets specific for each miRNA are shown in Tables 1 and 2. The SYBR green stem-loop RT-PCR method was used to assess the expression levels of the miRNAs. The PCR conditions were as follows: 95°C for 10 min, followed by 40 cycles of 95°C for 15 sec and 60°C for 1 min. Samples were run in duplicate with RNA preparations from three independent experiments. The reactions were conducted on the ABI PRISM 7900 system (Applied Biosystems). The fold change in the expression of each gene was calculated using the 2^−ΔΔ*CT*^ method, with U6 as an internal control.

### 2.9. Western Blot Analysis

H9c2 cells growing on six-well plates were transduced with miRNAs and treated with 400 *μ*M H_2_O_2_, as indicated. The proteins were separated on SDS-polyacrylamide gels and transferred to PVDF membranes. For immunoblotting, PVDF membranes were blocked and probed with antibodies overnight at 4°C. Immunocomplexes were visualized with horseradish peroxidase-coupled secondary antibodies.

### 2.10. Immunofluorescence Detection of Intracellular Cytochrome c Localization by Fluorescence Microscopy

After the appropriate treatment, the cells were washed with PBS and stained with 200 nM MitoTracker Red CMXRos dye (Molecular Probes, Inc., France), followed by incubation for 30 min at room temperature, to visualize the mitochondria. The cells were fixed with 4% paraformaldehyde for 15 min, permeabilized with 0.1% Triton X-100 for 10 min, and blocked using 3% serum dissolved in PBS for 30 min at room temperature. The cells were then probed with anti-cytochrome c antibody (1 : 40; Santa Cruz Biotechnology) overnight at 4°C. The cells were washed with PBS twice and incubated with FITC-conjugated secondary antibody (1 : 40; Biovision, China) for 2 h in the dark at 37°C. After washing, images of stained cells were obtained using a fluorescence microscope.

### 2.11. Statistical Analysis

All data are expressed as the mean ± SEM, unless indicated otherwise. Differences among groups were determined by ANOVA. Differences between groups were determined by Student's *t*-test, with *P* < 0.05 considered statistically significant.

## 3. Results

### 3.1. Effects of H_2_O_2_ on Cell Viability and Protein Expression

The viability of H9c2 cells was determined using the MTT assay by exposing the cells to different concentrations of H_2_O_2_ for 2 h. Although low concentrations of H_2_O_2_ had no effect on apoptosis and death, high concentrations (100–800 *μ*M) increased H9c2 cell death in a dose-dependent manner after a 2 h treatment under our experimental conditions (Figure 1(a)).

Because GPx1 is a major antioxidant enzyme that catalyzes the breakdown of H_2_O_2_, we hypothesized that exogenous H_2_O_2_ must induce endogenous Gpx1 expression changes in H9c2 cells. As shown in Figure 1(b), compared with untreated cells, a significant increase in GPx1 protein expression was observed in cells treated with H_2_O_2_ (100 and 200 *μ*M), suggesting that the exposure to moderate concentrations of H_2_O_2_ induces a compensation response, whereas 400 µM H_2_O_2_ damages the antioxidant enzyme system, resulting in decreased Gpx1 expression. Therefore, for the remainder of our experiments, a 400 *μ*M concentration of H_2_O_2_ was used to assess H_2_O_2_-mediated effects on H9c2 cells.

### 3.2. Predicted miR-181a as a Negative Regulator of Gpx1

To focus on the role of miRNAs as regulators of Gpx1, three commonly utilized miRNA target prediction algorithms (TargetScan, miRDB, and MiRanda) were interrogated for possible miRNAs interacting with Gpx1. The results of these three algorithms had four potential miRNA candidates in common: miR-7a, 125a, 181a, and 423 (Figure 2(a)). Next, to assess the expression of these candidate miRNAs induced by the apoptotic H_2_O_2_ concentration, H9c2 cells were exposed to 400 µM H_2_O_2 _for 2 h, and the expression levels of the miRNAs were determined by real-time PCR. If an miRNA candidate is a negative regulator of Gpx1, then H_2_O_2_ should increase its expression in H9c2 cells because the Gpx1 expression was downregulated after stimulation with 400 *μ*M H_2_O_2_ (Figure 1(b)). At the apoptotic concentration of H_2_O_2_, only miR-181a expression was increased compared with the control group, whereas the expression of the other candidate miRNAs was decreased (Figure 2(b)). To further confirm the expression change, a 2 h exposure of H9c2 cells to varying concentrations of H_2_O_2_ resulted in concentration-dependent increases in miR-181a expression, with a peak at approximately 400 *μ*M (Figure 2(b)). Taken together, these results suggest that miR-181a plays a key role in oxidative stress-induced cardiomyocyte apoptosis and that miR-181a may be linked with the expression of Gpx1.

### 3.3. Validation of the *In Silico* Target Analysis of miR-181a

To experimentally validate the computational data, a pmiR-RB-REPORT luciferase construct with the Gpx1-3′-UTR was generated. The purified gel product of Gpx13′-UTR was inserted into the cloning site downstream of the luciferase gene, as described in Section 2. A mutant version, pmiR-RB-Gpx1-3′-UTR-mut, with a three-base-pair mutation within the seed region (Figure 3(a)), was also generated. A significant decrease (*P < 0.01) in the relative luciferase activity was observed when the pmiR-RB-Gpx1-3′-UTR was cotransfected with a mature miR-181a into HEK293 cells compared with the miR-control. The miR-181a-mediated suppression was abolished by mutation of the 3′-UTR miR-181a binding site, which disrupts the interaction between miR-181a and the Gpx1-3′-UTR (Figure 3(b)).

Western blotting analyses further confirmed the luciferase assay results. The transfection with the mature miR-181a resulted in decreased Gpx1 protein expression (*P < 0.01) compared with the control, whereas the anti-miR-181a protected against the mature miR-181a-mediated inhibition of Gpx1 expression (*P < 0.05) (Figure 3(c)).

### 3.4. Transduction of the Anti-miR-181a Restored the H_2_O_2_-Altered H9c2 Cell Morphology and Decreased the Levels of LDH and MDA

H9c2 cells were transfected as described in Section 2. As shown in Figure 4(a), the mature miR-181a increased miR-181a expression in H9c2 cells, whereas anti-miR-181a decreased miR-181a expression. The control oligonucleotides had no effect on miR-181a expression.

H_2_O_2_ treatment changed the spindle-shaped, well-organized cell morphology into a shrunken, round, and distorted morphology. Transduction of the anti-miR-181a, however, almost restored the spindle-shaped morphology observed in untreated cells (Figure 4(b)). MDA levels are indicative of cardiomyocyte oxidativedamage. The H_2_O_2_ treatment strikingly increased the MDA level, whereas the miR-181a inhibitor significantly decreased the MDA level (Figure 4(c)). LDH release is an indicator of cellular injury. Compared with untreated cells, the LDH levels were markedly increased by H_2_O_2_-induced injuries. Transduction of the anti-miR-181a decreased LDH release, whereas transduction of the mature miR-181a elevated LDH levels compared with the miR-control (Figure 4(d)).

### 3.5. Anti-miR-181a Reduced ROS Production

Because Gpx1 catalyzes the reduction of H_2_O_2_ to water [5] and miR-181a mediates the suppression of Gpx1 expression, we attempted to investigate the effect of miR-181a upon ROS generation. ROS production was detected using an ROS-sensitive dye, 2′,7′-dichlorofluorescein-diacetate (DCFH-DA). As shown in Figure 5(a), H_2_O_2_ treatment led to strong DCFH-DA staining. Transduction of the mature miR-181a increased the staining intensity, whereas the anti-miR-181a produced relatively dim DCFH-DA staining. These data suggest that the anti-miR-181a attenuates the production of ROS. ROS production was quantified by measuring the cellular fluorescence intensities (Figure 5(b)).

### 3.6. Anti-miR-181a Attenuated H_2_O_2_-Induced H9c2 Cell Apoptosis

Compared with the control group, significantly more H_2_O_2_-treated cells underwent apoptosis, as shown by the bright DAPI staining in the H_2_O_2_ group.The H_2_O_2_ treatment caused nuclear condensation, an indicator of apoptosis. Transduction of the anti-miR-181a, however, nearly restored H9c2 nuclei to the normal morphology (Figure 6(a)). Quantitative analysis using flow cytometry confirmed that the anti-miR-181a significantly inhibited H_2_O_2_-induced apoptosis (Figures 6(b)-6(c)). To investigate the mechanism by which the anti-miR-181a attenuates the H_2_O_2_-induced H9c2 apoptosis, we examined the protein levels of Bcl-2 and Bax. Western blot analyses showed that Bcl-2 protein levels were markedly increased in the anti-miR-181a-treated cells compared with the miR-CTL group. As expected, Bax expression was markedly decreased by the anti-miR-181a (Figures 6(d) and 6(f)), suggesting that the anti-miR-181a prevents H9c2 cells from undergoing apoptosis by increasing Bcl-2 while inhibiting Bax.

### 3.7. Anti-miR-181a Restored the H_2_O_2_-Induced Loss of the Mitochondrial Membrane Potential

Untreated cells contained bright-staining mitochondria that emitted orange fluorescence. The H_2_O_2_ treatment caused the formation of monomeric JC-1, indicative of a loss of mitochondrial membrane potential. Transduction of the anti-miR-181a, however, blocked the H_2_O_2_-induced formation of JC-1 monomers (Figure 7(a)), suggesting that the anti-miR-181a can restore the H_2_O_2_-induced loss of the mitochondrial membrane potential. The ratio of orange to green fluorescence was used to quantify the Δ*ψ*m, with a low ratio representing mitochondrial depolarization. We found that the ratio of the H_2_O_2_ group was lower than that of the control group (*P < 0.01), that the anti-miR-181a showed protective effects compared with the anti-CTL-treated groups, and that the upregulation of miR-181a decreased the ratio (^&^ *P* < 0.05, ^#^ *P* < 0.05; Figure 7(b)).

### 3.8. Downregulation of miR-181a Blocks the Mitochondrial Apoptotic Pathway

The release of cytochrome c from the mitochondrial intermembrane space into the cytoplasm is a critical step in the progression of the intrinsic apoptotic pathway [19]. H_2_O_2_ treatment for 2 h increased the release of cytochrome c from the mitochondria, as shown by the loss of the colocalization of cytochrome c with the mitochondria (Figure 8). The effect of H_2_O_2_ was attenuated by transduction with the anti-miR-181a, whereas the upregulation of miR-181a exacerbated this effect (Figure 8).

Caspase-3 mediates apoptosis by regulating many important events that lead to the completion of apoptosis [20]. To further investigate the effects of mature miR-181a and anti-miR-181aon cleaved caspase-3 activation, we measured cleaved caspase-3 protein expression (Figures 6(d)-6(e)) by western blots in five different groups. The H_2_O_2 _treatment increased the generation of cleaved caspase-3. This effect was attenuated by transduction with the anti-miR-181a, whereas the upregulation of miR-181a increased cleaved caspase-3 expression (Figure 6(e)). These data suggest that the anti-miR-181a reduces H_2_O_2_-induced apoptosis by blocking caspase-3-dependent cardiomyocyte apoptosis.

## 4. Discussion

Increased ROS levels are a hallmark of oxidative stress-induced cardiomyocyte apoptosis. Compared with other ROS, H_2_O_2_ is a relatively long-lived molecule commonly used in models of oxidative stress in H9c2 cardiomyocytes [21, 22]. High concentrations of H_2_O_2_ (100–200 *μ*M) have been shown to increase apoptosis, whereas higher concentrations of H_2_O_2_ (300–1000 *μ*M) cause both apoptosis and necrosis in adult rat ventricular myocytes [23]. In our experiments, the treatment of H9c2 cells with H_2_O_2_ (50–800 µM) for 2 h caused a dose-dependent decrease in cell viability. A 400 µM dose of H_2_O_2_ induced both apoptosis and necrosis, as shown by flow cytometry. The dynamic oxidant/antioxidant balance is perturbed following the addition of exogenous H_2_O_2_ to the medium of cultured cells. In cultured neurons isolated from GPx1 knockout (GPx1^−/−^) mice, the susceptibility to H_2_O_2_-induced apoptosis correlates with the increasing accumulation of intracellular ROS [24]. We found that the levels of Gpx1 protein were significantly increased in cells exposed to 100 or 200 µM H_2_O_2_, suggesting that the exposure to moderate concentrations of H_2_O_2_ induces a compensation response, whereas 400 µM H_2_O_2_ damages the antioxidant enzymes system and leads to decreased Gpx1 expression.

miRNAs are endogenous regulators of gene expression. Previous reports have shown that the binding sites of target mRNAs with as few as seven complimentary base pairs (the seed sequence) to the miRNA 5′ end are sufficient for miRNA regulation in animals [25]. More recently, several studies indicated that miRNA expression levels were sensitive to H_2_O_2_ in cardiac myocytes. miRNAs can be used as powerful tools to modulate a functional phenotype that involves the participation of multiple proteins, as in the case of ROS-mediated events [26–29]. This finding raises the question of whether the oxidative stress-responsive miRNAs play a role in altering the expression of antioxidant genes that quench ROS to maintain redox homeostasis. With the help of current bioinformatics tools, we predicted several miRNAs that may target Gpx1. Although potential miRNAs can be predicted by computational analysis, these miRNAs must be experimentally verified in cells because the targets and functions of miRNAs are cell-specific and each single protein-coding gene can be regulated by multiple miRNAs [30, 31]. To test which miRNAs target Gpx1 mRNA in H9c2 cells, we first confirmed that the 400 µM H_2_O_2_ treatment decreased Gpx1 expression. Considering the negative relationship between miRs and Gpx1, the selected miRs were expected to be upregulated in H_2_O_2_-treated H9c2 cells. By qPCR analyses, we validated that the miR-181a expression was upregulated approximately 4-fold in H_2_O_2_-treated cells compared with the controls. In addition, Gpx1 expression in H9c2 cells was regulated by miR-181a in unstimulated cells, as determined both by gain-of-function and loss-of-function approaches. To further confirm this effect, we utilized a luciferase vector with the cloned target 3′-UTR region of Gpx1 mRNA. We demonstrated that the negative effect of miR-181a on the Gpx1 levels in H9c2 cells was the result of the direct targeting of Gpx1 mRNA by miR-181a. Hutchison et al. used microarray analysis to assess the effects of miR-181 on the transcriptome in primary astrocytes. Pathway and signaling pathway analyses demonstrated that miR-181 targets genes encoding antioxidant enzymes, including glutathione peroxidases 1 and 4 (Gpx1 and Gpx4, resp.) [32].

To ascertain the role of miR-181a in ROS-mediated H9c2 cells apoptosis, miR-181a expression was modulated via a miR-181a inhibitor and miR-181a mimic. ROS cause damage to intracellular macromolecules, including DNA breakage and lipid membrane peroxidation, both of which can be detected morphologically (cell shrinkage and nuclear condensation) and biochemically (DNA fragmentation and extracellular exposure of phosphatidylserine). We found that the downregulation of miR-181a expression protected against the H_2_O_2_-induced injury of H9c2 cells by restoring the alterations of H9c2 morphology and nuclear condensation, inhibiting the production of ROS and blocking LDH release and MDA production, two indicators of oxidative stress-induced injury [33].

The pivotal role of mitochondria in cell death and cell survival has been well established: mitochondrial dysfunction constitutes a critical event in the apoptotic process [34, 35]. Excessive levels of ROS damage mitochondria, induce the translocation of Bax and Bad, open the permeability transition pore (PTP), and, thus, lead to mitochondrial depolarization and outer membrane rupture, accompanied by the mitochondrial release of cytochrome c and late activation of caspase-3, finally causing cell apoptosis or death [19]. Our data demonstrate that the anti-miR-181a blocked H_2_O_2_-induced H9c2 apoptosis by regulating mitochondria-related apoptotic pathways. H_2_O_2_ induced a decrease in the mitochondrial membrane potential, suggesting an impairment of mitochondrial function. Transduction of the anti-miR-181a, however, restored the mitochondrial membrane potential. These data demonstrate that the anti-miR-181a protected H9c2 cells from H_2_O_2_-induced apoptosis by maintaining mitochondrial membrane integrity and cardiomyocyte function. Moreover, previous studies indicated that the Bcl-2 family is upregulated during the opening of the PTP [36]. Critical interactions between Bcl-2 family proteins cause permeabilization of the outer mitochondrial membrane, a common decision point early in the intrinsic apoptotic pathway that irreversibly commits the cell to death [37, 38]. Our results demonstrate that miR-181a regulates the expression of the Bcl-2 family. The anti-miR-181a significantly increased Bcl-2 levels while decreasing Bax protein levels, attenuating the alterations caused by H_2_O_2_-induced injury. One recent study demonstrated that cardiac mitochondria from GPx1^−/−^ mice lost their resistance to hypoxia/reoxygenation damage [39]. Previous studies have indicated that Bcl-2 knockout mice have reduced glutathione levels and glutathione peroxidase activity in brain tissue [40]. Other works have shown that GPx1 may modify the ratio of Bax to Bcl-2 to create a more antiapoptotic environment [41]. Therefore, it is reasonable to conclude that miR-181a regulates the expression of Gpx1 and that Gpx1 directly influences the expression of Bcl-2. However, the direct regulation of Bcl-2 by miR-181a has been confirmed by many investigations, mainly in tumor cells [42–44]. In the future, luciferase reporter assays and western blot analyses should be used to validate Bcl-2 as a direct target of miR-181a in H9c2 cells.

In addition to *cis*-regulation (direct targeting of mRNAs to induce degradation or inhibit protein translation), miRNAs may alter the expression of transcription factors or other regulatory genes that can affect the regulation of the target gene via *trans*-regulatory mechanisms [45]. Prior studies have identified several targets for miR-181a, including GRP78, a major endoplasmic reticulum chaperone and signaling regulator [46, 47], and sirtuin-1, an NAD-dependent protein deacetylase [48]. We assume that these targets may participate in the *trans*-regulation of Gpx1. Furthermore, other studies have demonstrated that miR-181a represses important antiapoptotic targets such as X-linked inhibitor of apoptosis (XIAP), a function that could help explain the proapoptotic effects of this miRNA [32].

In other studies, miRNAs have been shown to be directly linked to the regulation of antioxidant enzymes, including catalase [49], SOD_2_ [50], and NADPH oxidase [51]. Our study illustrates the role of miR-181a as a proapoptotic modulator in the regulation of Gpx1. Future studies, especially in ischemia/reperfusion animal models, are necessary to validate the possible therapeutic use of miR-181a regulation.

In summary, we have demonstrated that miR-181a expression is upregulated in H_2_O_2_-treated H9c2 cells and that inhibition of miR-181a confers cardiac protection against oxidative stress-induced H9c2 cell apoptosis through the direct inhibition of Gpx1 expression and ROS generation, which are important for the maintenance of mitochondrial membrane integrity and the inhibition of mitochondrial apoptotic pathway under oxidative stress conditions. These novel findings may have extensive diagnostic and therapeutic implications for a variety of cardiovascular diseases related to ROS, including atherosclerosis, hypertension, restenosis after angioplasty or bypass, diabetic vascular complications, and transplantation arteriopathy.

## Figures and Tables

**Figure 1:** Cell viability and protein expression changes in H_2_O_2_-treated H9c2 cells. (a) H9c2 cells were treated with various doses of H_2_O_2_ for 2 h and assessed for cell viability. *P < 0.05 versus control (CTL); **P < 0.01 versus control (CTL); the values represent the mean ± SEM, *n* = 5. (b) Gpx1 and *β*-actin protein levels were detected by western blotting after the treatment of H9c2 cells with different concentrations of H_2_O_2_ for 2 h. *P < 0.05 versus control (CTL); **P < 0.01 versus control (CTL); the values represent the mean ± SEM, *n* = 3.

**Figure 2:** miRNA expression changes in H_2_O_2_-induced apoptotic cardiomyocytes. (a) Fold change in miR-7a, 125a, 181a, and 423 expression after exposure to H_2_O_2_ (400 *μ*M) for 2 h. *P < 0.01 versus control (CTL); the values represent the mean ± SEM, *n* = 3. (b) H9c2 cells were treated with different concentrations of H_2_O_2_, ranging from 50 to 800 *μ*M for 2 h. *P < 0.05 versus control (CTL); **P < 0.01 versus control (CTL); the values represent the mean ± SEM, *n* = 3.

**Figure 3:** Gpx1 3′-UTR is a direct target of miR-181a. (a) Predicted miR-181a target site in the 3′-UTR of rat Gpx1. The wild-type rat Gpx1 mRNA sequence is shown with the potential binding sites. The mature miR-181a sequence and potential binding between the miR-181a seed region and the rat Gpx1 3′-UTR sequence are shown, with the mutated bases indicated above in red. (b) Rat Gpx1 3′-UTR reporter and the miR-181a binding site mutant reporter were cotransfected with either the mature miR-181a (50 nM) or miR-CTL into HEK 293T cells, followed by cell lysis and luciferase assays 48 h later. *P < 0.01 versus Gpx1-WT+miR-CTL group; the values represent the mean ± SEM, *n* = 3. (c) Gpx1 and *β*-actin protein levels were detected by western blotting 48 h after H9c2 cells were transfected with miR-CTL, miR-181a (50 nM), anti-CTL, or anti-miR-181a (100 nM). *P < 0.01 versus miR-CTL; ^&^ *P* < 0.01 versus anti-CTL group; the values represent the mean ± SEM; *n* = 3.

**Figure 4:** Effects of the down- or upregulation of miR-181a on H_2_O_2_-induced H9c2 cell morphology and cellular injury. H9c2 cardiomyocytes were treated with miRNAs for 6 h prior to H_2_O_2_ (400 *μ*M, 2 h) treatment. (a) H9c2 cells were transfected with miR-CTL, miR-181a (50 nM), anti-CTL, or anti-miR-181a (100 nM) for 6 h, followed by real-time PCR analysis of the miR-181a expression levels 24 h later. *P < 0.01 versus miR-CTL; ^&^ *P* < 0.01 versus anti-CTL group; the values represent the mean ± SEM; *n* = 3. (b) The downregulation of miR-181a restored the oxidative stress-induced alteration of H9c2 cell morphology, whereas the upregulation of miR-181a exacerbated the morphological changes. Scale bar: 25 *μ*m. (c) The cellular MDA levels were measured using the TBA method, and the concentration of MDA was expressed as nmol/mg protein. *P < 0.01 versus control (CTL); ^&^ *P* < 0.01 versus miR-CTL; ^#^ *P* < 0.01 versus anti-CTL group; the values represent the mean ± SEM; *n* = 5. (d) The LDH activity in the culture medium was measured, and the results are expressed as U/L. *P < 0.01 versus control (CTL); ^&^ *P* < 0.01 versus miR-CTL; ^#^ *P* < 0.01 versus anti-CTL group; the values represent the mean ± SEM; *n* = 5.

**Figure 5:** Effects of the miR-181a and anti-miR-181a on H_2_O_2_-induced H9c2 cell ROS generation. (a) The intracellular ROS levels were estimated using the probe DCFH-DA. ROS production was observed using a fluorescence microscope. (b) The ROS production was quantified by a fluorescence microplate reader, with the fluorescence read at 485 nm for excitation and 530 nm for emission. The cellular fluorescence intensities were expressed as the multiple of the level in the control group. *P < 0.01 versus control (CTL); ^&^ *P* < 0.01 versus miR-CTL; ^#^ *P* < 0.01 versus anti-CTL group; the values represent the mean ± SEM; *n* = 5.

**Figure 6:** Effects of the miR-181a and anti-miR-181a on H_2_O_2_-induced H9c2 cell apoptosis and the expression levels of key mediators of apoptosis. The cells were transfected with miRNAs for 6 h and cultured for 24 h, with H_2_O_2_ (400 *μ*M) added for the last 2 h. (a) Oxidative stress-induced DNA damage in the nuclei was shown by DAPI staining. ((b)-(c)) H9c2 cell apoptosis due to oxidative stress was analyzed by flow cytometry. *P < 0.01 versus control (CTL); ^&^ *P* < 0.01 versus miR-CTL; ^#^ *P* < 0.01 versus anti-CTL group; the values represent the mean ± SEM; *n* = 5. (d) The cleaved caspase-3, Bcl-2, and Bax protein levels were detected by western blot. (e) The normalization of cleaved caspase-3 expression to that of *β*-actin. *P < 0.01 versus miR-CTL; ^&^ *P* < 0.01 versus anti-CTL group; the values represent the mean ± SEM; *n* = 3. (f) Bcl2/Bax ratio. *P < 0.01 versus miR-CTL; ^&^ *P* < 0.01 versus anti-CTL group; the values represent the mean ± SEM; *n* = 3.

**Figure 7:** Effects of the miR-181a and anti-miR-181a on the H_2_O_2_-induced reduction of the mitochondrial membrane potential. (a) The mitochondrial membrane potential was assessed by the lipophilic cationic probe JC-1. An orange signal indicates the aggregation of JC-1 in the mitochondria. A green signal represents cytosolic JC-1 monomers, indicative of the loss of the mitochondrial membrane potential. Merged images show the colocalization of the JC-1 aggregates and monomers. Scale bar: 25 *μ*m. (b) Quantitative analysis of the membrane potential in (a). The Δ*ψ*m of the H9c2 cardiomyocytes in each group was calculated as the ratio of orange to green fluorescence, expressed as the multiple of the level in the control group. *P < 0.05 versus control (CTL); ^&^ *P* < 0.05 versus miR-CTL; ^#^ *P* < 0.05 versus anti-CTL group; the values represent the mean ± SEM, *n* = 3.

**Figure 8:** Effects of the miR-181a and anti-miR-181a on H_2_O_2_-induced cytochrome c release from the mitochondria in H9c2 cells. Fluorescence microscopy analysis of H9c2 cells transfected with miRNAs for 6 h prior to exposure to H_2_O_2_ (400 *μ*M) for 2 h shows immunostaining of cytochrome c (green), Mito tracker staining of the mitochondria (red) and merged images of the two, showing colocalization in yellow. Upon the release of cytochrome c from the mitochondria, green fluorescence can be seen independently. Scale bar: 25 *μ*m. The images presented are representative of three independent experiments.

**Table 1:** Sequences of the RT primers.

Primer name	RT primer sequence
U6	5′CGCTTCACGAATTTGCGTGTCAT3′
rno-miR-7a	5′GTCGTATCCAGTGCGTGTCGTGGAGTCGGCAATTGCACTGGATACGACACAACAA3′
rno-miR-181a	5′GTCGTATCCAGTGCGTGTCGTGGAGTCGGCAATTGCACTGGATACGACCATGGA3′
rno-miR-125a	5′GTCGTATCCAGTGCGTGTCGTGGAGTCGGCAATTGCACTGGATACGACTCACAGG3′
rno-miR-423	5′GTCGTATCCAGTGCGTGTCGTGGAGTCGGCAATTGCACTGGATACGACACTGAGG3′

**Table 2:** Sequences of the primers used in the SYBR-green-based quantitative RT-PCR validation.

Primer name	Primer sequence	Tm (°C)	Length (bp)
U6	F: 5′GCTTCGGCAGCACATATACTAAAAT3′	60	89
	R: 5′CGCTTCACGAATTTGCGTGTCAT3′		

rno-miR-423	F: 5′TAAGCTCGGTCTGAGGC3′	60	65
	R: 5′CAGTGCGTGTCGTGGA3′		

rno-miR-7a	F: 5′GGGGTGGAAGACTAGTGATT3′	60	67
	R: 5′CAGTGCGTGTCGTGGA3′		

rno-miR-181a	F: 5′GGGCAGCCTTAAGAGGA3′	60	64
	R: 5′CAGTGCGTGTCGTGGA3′		

rno-miR-125a	F: 5′GCTCCCTGTAGACCCTTTA3′	60	67
	R: 5′CAGTGCGTGTCGTGGAGT3′		
